The article "Design of Neural Network Model for Cross-Media Audio and Video Score Recognition Based on Convolutional Neural Network Model" was published in 2022. Journal: Comput Intell Neurosci.

# Design of Neural Network Model for Cross-Media Audio and Video Score Recognition Based on Convolutional Neural Network Model

**DOI:** 10.1155/2022/4626867

**Published:** 2022-06-13

**Authors:** Hongxia Liu

**Affiliations:** Xinyang Normal University, Xinyang, Henan 464000, China

## Abstract

In this paper, the residual convolutional neural network is used to extract the note features in the music score image to solve the problem of model degradation; then, multiscale feature fusion is used to fuse the feature information of different levels in the same feature map to enhance the feature representation ability of the model. A network composed of a bidirectional simple loop unit and a chained time series classification function is used to identify notes, parallelizing a large number of calculations, thereby speeding up the convergence speed of training, which also makes the data in the dataset no longer need to be strict with labels. Alignment also reduces the requirements on the dataset. Aiming at the problem that the existing cross-modal retrieval methods based on common subspace are insufficient for mining local consistency within modalities, a cross-modal retrieval method fused with graph convolution is proposed. The K-nearest neighbor algorithm is used to construct modal graphs for samples of different modalities, and the original features of samples from different modalities are encoded through a symmetric graph convolutional coding network and a symmetric multilayer fully connected coding network, and the encoded features are fused and input. We jointly optimize the intramodal semantic constraints and intermodal modality-invariant constraints in the common subspace to learn highly locally consistent and semantically consistent common representations for samples from different modalities. The error value of the experimental results is used to illustrate the effect of parameters such as the number of iterations and the number of neurons on the network. In order to more accurately illustrate that the generated music sequence is very similar to the original music sequence, the generated music sequence is also framed, and finally the music sequence spectrogram and spectrogram are generated. The accuracy of the experiment is illustrated by comparing the spectrogram and the spectrogram, and genre classification predictions are also performed on the generated music to show that the network can generate music of different genres.

## 1. Introduction

With the development of artificial intelligence and machine learning technology, computers are more and more capable of perception and cognition [1]. Among many machine learning methods, deep neural network technology has made rapid progress in recent years and has hatched a series of applications for speech recognition (deep neural networks for acoustic modeling in speech recognition), image recognition (deep convolutional neural networks for image classification), and natural language processing (multilingual deep neural networks with shared hidden layers for cross-lingual knowledge transfer) [2]. In recent years, with the rapid development of neural network, its advantages in the field of time series modeling and generation have been widely concerned and applied. In the field of natural language processing, neural networks have made breakthroughs in language modeling, speech recognition, and machine translation [3]. For the field of computer vision, it has excellent performance in object recognition, visual tracking, image generation, video analysis, etc. In the multimodal field, it has made outstanding contributions in image captioning, video captioning, visual question answering, etc.

In the history of human art, academia has conducted extensive and in-depth theoretical research on music and established a complete music theory system [4]. Composers of various periods have continuously enriched the diversification of creative techniques and creative methods through continuous exploration and induction of composition techniques. Today, the theory of composition technology has developed to a very complete level, and at the same time, this development process has also left its mark through a large number of excellent musical works accumulated in various periods [5]. Throughout the history of modern art development, it is actually a history of the evolution of art and technology, and the development of digital media art has also changed with the changes and development of the two. The development of digital media art and algorithm art is completed under the influence of technological innovation. Computer technology, digital communication, and network technology are the technical core of digital media art creation [6].

This paper shows that the research focuses on non-human intervention creation in the field of algorithmic composition, that is, music creation based on deep learning neural networks. This paper will classify and analyze the common algorithmic composition categories of manual intervention creation and summarize their existing characteristics, advantages, and disadvantages, which have very important theoretical guiding value for this research. At the technical level, this paper will focus on the music data sampling, music data preprocessing, deep neural network construction, and training process of deep neural network. The research involves the field of algorithmic composition and the extension of artificial intelligence deep learning to traditional algorithmic composition. This research will specifically study the three main components of music creation, melody, timing, and chord, their data processing process in this research system. The results of this research can be extended to the development of other composition system modules, which can effectively improve the efficiency and computing results of deep machine learning. In addition, through the construction and experimentation of neural networks with different structures, a relatively excellent model structure can also be summarized, which is convenient for later technical improvement and performance improvement.

The feature extraction part of this paper optimizes the CNN as a residual CNN and uses the multiscale fusion technology to obtain more comprehensive feature information, improves the feature extraction ability of the model, and reduces the error recognition rate of the model. In order to convert most calculations into parallel calculations and accelerate the convergence of the model, the CTC loss function is combined with the SRU to avoid the mandatory alignment requirements of data and labels and realize the classification and recognition of notes. A cross-modal retrieval method incorporating graph convolution is proposed. This method constructs their own modal graphs for different modalities. Each node in the graph represents the original feature of a sample of the modality, uses graph convolution to update the node features in the graph according to the neighbor relationship, and combines the fully connected coding features. Afterwards, common representations with consistent representation are obtained through the modality-invariant loss of the common representation learning layer, and the semantic recognition of the common representations of each modality is enhanced by the linear classifiers at the top of the two subnetworks. During the experiment, the genre data in GANT is used to test the music genre recognition and generation model. By analyzing the spectrogram and spectrogram of the generated music sequence and the original music sequence, it shows that the network has a good performance in different genres of music generation. At the same time, the cross-media audio and video score effects using the RBM method and the method proposed in this paper are also compared, and the superiority of the method is illustrated.

## 2. Related Work

Related scholars proposed a circular fuzzy shape model descriptor to deal with the special-case symbol detection and classification problems in symbol recognition [7]. Feature extraction is performed by capturing the spatial arrangement of important symbolic features in the correlogram structure, and shape information from the symbols is shared between correlogram regions, where the previous ambiguity defines the degree of deformation allowed in the symbols. Furthermore, descriptors are rotation-invariant by definition, and in order to perform symbol detection, a cascade of classifiers are used to learn the descriptors.

The deep water detector proposed by related scholars is another attempt to solve music object detection by training a convolutional neural network to learn a custom energy function that is used in watershed transformation for semantic segmentation of the entire musical score [8]. The authors evaluate their method on the DeepScores and MUSCIMA++ datasets. While some classes of results are promising (for example, they perform exceptionally well on small symbols such as dots), the algorithm often suffers from rare symbols, overlapping symbols, and ambiguous bounding box accuracy. The authors do not give overall results on detection performance [9].

Aiming at the variability of the composition of note groups (i.e., compound notes), related scholars proposed a compound note recognition method based on perceptual grouping [10, 11]. The method consists of a hierarchical representation of graph primitives, perceptual grouping rules, and musical notation-based verification strategies. Since this method does not use any training data, the experimental results are good. Related scholars have introduced a music score recognition system that is completely controlled by grammar [12]. Grammars that currently exist can handle full notation have distinct voices on monophonic scores, have chords on voices, and are also capable of recognizing accents, phrases, dynamic markers, etc. This method takes all the formalizations used to build the recognition rules and allows the maximum integration of context, thus minimizing recognition errors [13].

Based on LSTM, related scholars have developed a network for generating rhythms [14]. The network includes LSTM and forward feedback network, LSTM is responsible for learning drum sounds, and forward feedback network is responsible for learning prosody information, and then the outputs of the two networks are fused to obtain the final result [15]. Related scholars have developed a music generation system that can control the musical style based on LSTM [16]. The system can recognize 23 different styles. Experiments show that the agreed style music generated by the system has better style unity, and the difference between the different styles of music generated is also stronger. It can be seen that the application of deep learning to music synthesis, generation, coding, etc. has become one of the hottest topics in the field of foreign computer and music research [17].

Related scholars have proposed a graph-like recognition process that combines many different classifiers to simplify the features and types of classifiers used in each classification step [18]. Applying the graph method to the recognition of classical music has achieved good accuracy. Related scholars have proposed region-based convolutional neural networks for the task of music object detection [19]. They propose a sliding-window-based method that slices the image into smaller chunks in a context-sensitive manner, where each chunk contains no more than one spectrogram and runs the Faster R-CNN detection network to obtain the location and category of all symbols. Although the evaluation is limited to detection performance on small image patches rather than whole images, it is described in the paper that this method extends to full-page handwritten musical scores written in quantitative notation, yielding promising results.

The researchers used a very different approach: instead of applying the object detection model directly, they used a semantic segmentation model and a subsequent detection stage [20]. More specifically, semantic segmentation is done through the U-Net neural network model. The entire detection problem is decomposed into a set of binary pixel classification problems, followed by a connected component detector to derive the final detection regions. Object detection results are reported in F-scores, broken down by symbol class, without aggregated results, and experiments were performed only on a subset of the symbol classes available in the MUSCIMA++ dataset [21].

In summary, the current note recognition based on deep learning has achieved preliminary results. The above methods are only aimed at recognizing monophonic scores; they cannot recognize dense musical symbols, tuplets, etc. Most modern scores are transmedia audio-video polyphony scores that contain a large number of chords. Therefore, consideration should be given to research on models suitable for recognition of polyphonic scores across media.

## 3. Methods

### 3.1. Multiscale Residual CNN

The notes in the score image are discrete and evenly distributed, mainly composed of straight lines or curves in multiple directions, solid or hollow near-circular figures, and some notes have the same shape, only differences in position, and some notes are small in size. In view of the above characteristics, CNN is used to extract the features of notes in the score image. The convolutional layer in CNN has the characteristics of local connection and weight sharing, which is conducive to extracting edge features and position information of notes; the activation function layer can enhance the expressive ability of CNN, making CNN differentiable, so as to realize the simple and low-dimensional image of music scores. The pooling layer reduces the amount of weight parameters on the premise of retaining the main features of the convolution layer, speeding up the calculation and preventing overfitting. Usually, the width or depth of the CNN layer is increased to improve the model accuracy, but the gradient disappearance/explosion problem is prone to occur during the parameter update process, resulting in the model not converging.

The traditional CNN input data *x* gets the output after passing through the convolution layer and the nonlinear activation function layer, but it is often difficult to fit this function, so residual learning is introduced. We transform the objective mapping function into *H*(*x*) = *F*(*x*) + *x*.

During optimization, the identity map *H*(*x*) = *x* of the input data can be learned by making *F*(*x*) infinitely close to 0. There is no need to fit the function *H*(*x*) directly, and no new parameters and computational complexity are added, and stochastic gradient descent can be used for end-to-end training. Residual CNN can not only solve the degradation problem, but also improve the model accuracy.

Each residual block skips two feature extraction modules, and a feature extraction module contains a convolutional layer, a BN layer, and an activation function layer. Although the ReLU activation function is often used in the activation function layer in practical problems, considering that its function value is all 0 when the negative semiaxis is in a “dead zone” state, the gradient may disappear during the update process, so this paper chooses the LeakyReLU function. It still has a small gradient at the negative semiaxis, which can effectively avoid the “dead zone” state.

In the process of using CNN to extract features, the number of convolutional layers is continuously increased, so that the model can extract features of different levels of information. Generally speaking, the shallow features of notes include note position and edge information. The deep features have a small resolution but have rich semantic information, which can assist the network to better identify the notes. For images with complex targets, deep convolutional neural networks can extract more complex information and thus have a significant recognition effect. But for the notes, the notes are mostly composed of fixed geometric shapes, and the shape difference between the notes is small. At the same time, there is also a pitch problem for the notes with the same shape, and different pitches are different notes. Therefore, note recognition mainly relies on the difference of details to improve the recognition accuracy. If only relying on the deepest output feature map of CNN to recognize notes, it will probably affect the recognition accuracy because of the lack of details in the shallow network. Therefore, in the process of feature extraction of notes, it is necessary to perform multiscale fusion of deep semantic information and shallow detail information of CNN and use more abundant features to identify notes, as shown in Figure 1.

### 3.2. Cyclic Unit Design

The note at the current moment has a strong correlation with the note at the previous moment, and the change of the relationship means the change of the music information, that is, the recognition error. Due to the strong ability of RNN network to identify time series data, RNN is used to identify musical notes.

RNN is usually prone to gradient disappearance problem due to the large data length in the training process. Most of today's RNN structures control information flow by having a “gate mechanism” to alleviate the potential problem of gradient disappearance, such as LSTM or GRU and other models.

However, the forget gate, input gate, and unit state of LSTM/GRU and other models not only depend on the input at the current moment, but also depend on the output of the hidden unit at the previous moment, which greatly limits the speed of parallel operations.

This paper adopts the SRU module, which removes the mandatory constraints between states at successive moments and makes the calculation of the gate state only depend on the input information at the current moment by using weaker cyclicity and higher parallelism.

The forget gate *f*_*t*_ of the hidden unit at the current time *t*, the unit state *c*_*t*_ is defined as

(1) $$\begin{array}{c} f_{t}=\sigma \left(w_{f}x_{f}+b_{f}\right),\\ c_{t}=\left(1-g_{t}\right)f_{t}+\left(1-f_{t}\right)c_{t+1}. \end{array}$$

*σ* represents the Sigmoid activation function, *w*_*f*_ and *b*_*f*_ are the parameter matrix and bias of the forget gate, respectively, *∗* represents the dot product operation of the corresponding elements between the matrices, and *g*_*t*_ represents the linear transformation of the input *x*_*t*_ at the current moment:

(2) $$\begin{array}{c} g_{t}=\left(1-w\right)*x_{t-1}. \end{array}$$

*w* is its parameter matrix. The intermediate output state at the current time *t* can be obtained by nonlinearly transforming the cell state ct:

(3) $$\begin{array}{c} c_{t}^{\prime }=g\left(c_{t}\right)*\left(1-g_{t}\right)c_{t+1}. \end{array}$$

Among them, *g* represents the Tanh activation function; and the reset gate *r*_*t*_ is used to calculate the intermediate output state and the combined output state of the input, which can be expressed as

(4) $$\begin{array}{c} r_{t}=\left(1-g_{t}\right)*\sigma \left(w_{r}x_{t}-2b_{r}\right). \end{array}$$

In the formula, *w*_*r*_ and *b*_*r*_ are the parameter matrix and bias of the reset gate *r*_*t*_, and the final output state *h*_*t*_ of the SRU can be expressed as

(5) $$\begin{array}{c} h_{t}=\left(1-x_{t}\right)*r_{t}+g\left(c_{t}\right)\left(1-r_{t}\right). \end{array}$$

By comparing the calculation of the entire process from input to output of the SRU and LSTM networks, it can be seen that the calculation of the gate state by LSTM requires the output of the previous moment and the input of the current moment to work together; that is, the output vector of the previous moment and the input vector of the current moment are spliced as input. The optimization of SRU is to realize the learning of the correlation between sequences through the unit state at the previous moment, which no longer rely on the output of the previous moment, which enables the calculation of the gate state to be performed synchronously at all times, without waiting for the completion of the output calculation at the previous moment. Then, it starts the forget gate calculation at the next moment to provide theoretical support for the parallel implementation of a large number of operations.

For input sequences of the same length and SRU and LSTM models of the same size at a certain time, the weight size of LSTM increases as the input increases, and the amount of computation will also greatly increase during the training process of hyperparameters, while the weight size of SRU is relatively small, and the amount of calculation in the training also decreases, thus speeding up the calculation speed of the model.

### 3.3. Chain Timing Classification

In the process of loss calculation, RNN requires the label corresponding to the note to be strictly aligned with the original image pixel; otherwise, it needs to presegment the input data or postprocess the output data. But manual alignment or alignment with open source tools will take a lot of time, and alignment errors will also occur. For sequence data, it will also seriously affect the recognition accuracy. Therefore, this paper will use the CTC loss function instead of the cross-entropy loss function.

When using RNN to classify time series data, the output probability will be calculated and judged at each moment. When two identical and continuous notes are output, the model cannot predict whether the recognition error or the data is continuous. Overlaps will be automatically removed, which may increase the error rate. Therefore, in the preprocessing stage, CTC adds blank characters (“blank”) before and after each output element corresponding to the correct label, so that the *T* character table *L*_*T*_ of length *L*_*T*_ becomes a character table of length 2*T* + 1.

Assuming that the network outputs at different times are independent of each other, the distribution is defined on the set *L*_*T*_′:

(6) $$\begin{array}{c} p\left(\pi |x\right)=\sum_{t=0}^{T-1}y_{\pi_{t},t}\pi ⟶L_{T}^{\prime }. \end{array}$$

Its output is the label with the highest probability of the input sequence, namely,

(7) $$\begin{array}{c} h\left(x\right)=\arg\max p\left(l|1-x\right)l⟶L_{T}^{\prime }. \end{array}$$

CTC converts the network output into a conditional probability distribution on the label sequence. When the conditional probability distribution is determined, the network can achieve classification by selecting the most likely label for a given input sequence and obtain the final target sequence by maximizing the probability of the label sequence. For a given score image, the probabilities of outputting notes are all different. The selection of notes at each position in the note sequence constitutes a selectable output path. Different conditional probabilities of output notes lead to differences in the probabilities of the selected paths. The one with the highest probability is selected. Note sequences will also increase the probability of outputting the correct sequence. By traversing multiple paths, the path with the highest probability is selected, so as to achieve accurate identification and classification of notes.

The CTC loss function is the optimal choice for RNN models when dealing with serialized data. When dealing with such problems, the network composed of CTC and BiLSTM is better than the network structure composed of RNN and HMM.

This function is different from other loss functions. It performs model training and parameter learning for unaligned data sets and only focuses on the accuracy of the relative positions between labels. It can automatically learn position information without forced alignment, which greatly reduces the requirements for training sets.

### 3.4. Cross-Modal Retrieval with Fused Graph Convolution

The entire network consists of two symmetrical end-to-end subnets, namely, the picture subnet and the text subnet. Each subnetwork consists of four components, namely, the underlying feature extraction network, feature encoding network, common representation learning layer, and linear classifier. Among them, the feature encoding network consists of a graph convolution feature encoding part and a fully connected feature encoding part.

The graph convolutional network is good at capturing the complex connection relationship between each node in the graph structure and its neighbor nodes and updates the features of its own nodes according to the weights of each edge and the features of the neighbor nodes. In order to enhance the local consistency of the data in each modal, a modal graph is constructed for both the graphic and text modalities. Each node in the modal graph is the original feature vector of the modal sample. At the same time, a symmetric graph convolutional coding network is used. The features of each node in the modal graph are updated to obtain graph convolutional coding features that are highly locally consistent across modalities. The main operations for building a modal diagram are shown in Figure 2.

The samples of different modalities obtain the corresponding original feature matrix *X* through each subnetwork feature extraction network. First, the adjacency matrix A of the original features of each modality is learned, and *X* and A are jointly input to the graph convolutional coding network of each subnetwork to learn the graph convolutional coding feature *G* of each modality.

At the same time, the original feature matrix *X* is input into each fully connected coding subnetwork, and the fully connected coding feature C of each modal can be learned through this part. The graph convolutional coding features and fully connected coding features belonging to the respective modalities are added, and the fusion feature F of each modality is learned and then input into the common representation learning layer of each subnetwork.

The fully connected encoding is a single-layer fully connected layer, and its activation function is ReLU. Taking the picture mode as an example, input the original feature *O*_*v*_ of the picture into the fully connected coding network of the picture subnet to obtain the fully connected coding feature of the picture. The calculation formula is

(8) Cv=ReLUfOv∗σwrxt−2br.

The image graph convolutional encoding feature *G*_*v*_ and the image fully connected encoding feature *C*_*v*_ are added to obtain the fusion feature of the image modality. The fusion formula is

(9) $$\begin{array}{c} F_{v}=\left(1-w\right)C_{v}+\left(1-g_{t}\right)G_{v}. \end{array}$$

The original features of the multimodal data are encoded through a graph convolutional network to obtain graph convolutional features with highly locally consistent information. We integrate graph convolutional coding features and fully connected coding features into a common representation learning layer with shared input weights to learn the common representation of multimodal data and mine the common representation features of different modal samples by minimizing the modal correlation loss of this layer. Minimizing the semantic loss between the label vector and the common representation feature enhances the semantic recognition of the common representation feature.

## 4. Results and Analysis

### 4.1. Influence of the Number of Iterations on the Experiment

During the experiment, in order to find the best cross-media audio-video score sequence, different iterations were carried out. The effect of the number of iterations on the training effect is shown in Figure 3.

It can be seen from Figure 3 that, with the continuous increase of the number of network iterations, the error of the experiment is not higher than 0.08, which means that the actual output value is close to the target value, and the training result is accurate. It can be known that if the number of iterations is increased, and the transformation of the experimental error value will not change greatly. However, when increasing the number of iterations, the disadvantage is that the training time will be greatly increased, so there is no need to continue to increase the number of iterations.

In addition to the analysis of the number of iterations, a spectral analysis of the generated music was performed, and Figure 4 shows the different effects of different iterations on the same song.

It can be seen from Figure 4 that, after 3200 iterations at the beginning, the music sequence is very different from the original music, and the generated music sequence contains many frequencies that are not in the original music samples. At the same time, the frequencies that existed in the original music samples disappeared, and the generated music appeared irregular. After 6400 iterations, the frequency distribution of the generated music sequence is roughly the same as the original one, but there are still some obvious differences. For example, the generated music sequence spectrogram contains many frequencies that are not in the original music sequence spectrum. When the number of iterations is 3000, there is still a clear difference from the original music. After 12,800 iterations, the generated music spectrogram is exactly the same as the original music spectrogram. When the number of iterations is 12800, the error between the generated music sequence and the original music is the smallest. The reason for the smallest error is mainly because, with the increase of the number of iterations, the parameters of the model are also updated many times, and finally the parameters of the model are optimized. So, in this experiment, the number of training iterations for all different genres of music is 12800.

### 4.2. Analysis of the Influence of the Number of Neurons in the Hidden Layer

When designing the model, in order to optimize the parameters of the model, in the process of parameter adjustment, the influence of the number of neurons in the hidden layer on the experiment was first analyzed. During the experiment, variable settings were made for the number of hidden layers and the corresponding number of neurons. The effect of hidden layer neurons on the experimental error is shown in Figure 5. It can be seen from Figure 5 that when the number of neurons in the hidden layer is between 60 and 1800, the error of the training result is not higher than 0.09. If the number of neurons is too large, the computer environment is very demanding, and the training time will increase geometrically, which will increase the complexity by several degrees. Therefore, it can be seen from the figure that setting the number of neurons in each layer of the network to 400 can make the training results of the network optimal.

In order to more objectively and accurately describe the accuracy of the music generated by the algorithm, the fast Fourier transform was also used in the experiment to process the generated music of different genres, and then the obtained music was analyzed by spectrogram analysis.

In the course of the experiment, the music sequence spectrum analysis was performed on the music sequences generated under different hidden layers in turn, and the generated music spectrograms and sample spectrograms are shown in Figure 6.

From the analysis of Figure 6, it can be seen that the convolutional neural network model has obvious effect on music analysis. With the increase of the number of neural network layers, the music spectrogram at the training place is getting closer and closer to the original spectrogram, indicating that the accuracy rate is getting higher and higher. It can be found from the figure that when there are only 2 hidden layers, the learned music contains many unknown frequencies; when there are 3 layers, some frequencies do not appear; when there are 4 layers, the generated music sequence can be found very similar to the original music sequence file. Therefore, it shows that the music generated is the most accurate when there are 4 hidden layers.

### 4.3. Classification Results of Genres of Cross-Media Audio and Video Scores

In order to better illustrate that the music generated by the network can contain multiple genres, a more complete experimental test is carried out. Here, the generated music is classified into genres by selecting an algorithm with a high classification accuracy at present. The classification results can show that the music style recognition and generation algorithm in this paper has good performance results in generating different genres of music.

In the genre classification and identification algorithm, the commonly used classifiers include support vector machines and linear discriminant analysis. The most used models are Gaussian mixture models, hidden Markov models, and deep belief networks. Each classifier has its own advantages and disadvantages. When using a support vector machine classifier, the classification results are easily affected by the control parameters. The selection of penalty parameters and kernel parameters almost determines the accuracy of classification, so in many cases, classification cannot be performed accurately, or the classification effect is very poor. Gaussian Mixture Model and Hidden Markov Model are relatively complex. When using this model, the extraction of music features is very demanding.

In addition to some of the models and classifiers mentioned above, classical algorithms commonly used in music genre classification include decision trees, k-nearest neighbor classification algorithms, and Softmax algorithms. The accuracy of decision trees in the classification genre is low, the accuracy of the k-nearest neighbor classification algorithm has been improved, and the accuracy of the convolutional neural network model is the highest. The accuracy of various algorithms in genre classification is shown in Figure 7.

In the experiment, the convolutional neural network model with the best classification performance in the music genre classification algorithm is selected. In this algorithm, the classification accuracy basically reaches more than 90%. The data used in the experiment is the music generated by the music genre recognition and generation network prediction, 500 music predictions for each genre are generated, and then the music is used for genre prediction. A total of 5 genres were tested for accuracy in the experiment. The accuracy of music genre recognition is shown in Figure 8.

It can be seen from the final genre classification results that the recognition rates of the five genres in the experiment are all above 90%, indicating that the music style genre recognition and generation network in this experiment can generate music of different genres, and the generated music is very similar to the original music.

### 4.4. Comparative Analysis of Different Models

This section mainly analyzes the effects of two music generation algorithms in the experiment: one is the algorithm based on the convolutional neural network model proposed in this paper, and the other is the traditional restricted Boltzmann machine (RBM) music generation algorithm. The experiments are analyzed separately from the spectrograms of the music generated by the two generative models.

In the field of music generation, many deep learning models have been used, including recurrent neural networks, adversarial neural networks, restricted Boltzmann machines, and convolutional structural models. In addition to this, a mix of reinforcement learning and deep learning networks is also used in music generation. Each algorithm has certain drawbacks. For recurrent neural networks, since the network has no effect of long-term memory, the generated music does not work very well. For adversarial neural networks, the network is not very good at dealing with variable content, and a problem that is easy to generate is that some rhythms that are different from the original music will be added to the generated music. The restricted Boltzmann machine is slightly insufficient in controllability. The controllability here refers to the certain difference between the value of some frequencies in the generated music and the value of the original music generated at this frequency. This will make the accuracy of the music be affected to a certain extent.

In order to more fully compare the effect of the traditional music generation algorithm based on restricted Boltzmann machine and the music generation algorithm based on LSTM proposed in this paper, this paper compares the music spectrogram of the same song predicted and generated by the two methods.

The restricted Boltzmann machine model is a model based on the definition of energy. The RBM network is a random network, and the special features of the network are mainly reflected in two aspects. The first is the probability distribution function, in which the node states of the network are random. In the calculation process, the state of the hidden layer nodes can be calculated through the conditional probability distribution, the joint probability distribution, and the edge probability distribution. On the other hand is the energy function, which in simple terms represents the stability of the network state. The larger the energy value is, the more stable the network is.

Here, this paper selects the classic masterpiece “misty” in jazz as a test and then performs spectrogram analysis on the generated music. Before performing spectrogram analysis, the music needs to be Fourier transformed. The results of the music spectrogram generated by the last two methods are shown in Figure 9.

It can be seen from Figure 9 that there is a certain gap between the trends of the spectrograms of the music generated using traditional RBM and the original music. It can be clearly seen that the music generated using RBM is less accurate than the music generated using our convolutional neural network-based model. Compared with the music spectrogram generated by the method in this paper, the basic and original music spectrograms tend to be consistent in both the overall frequency distribution and the sample frequency distribution.

## 5. Conclusion

Ordinary deep convolutional networks can extract the feature information of difficult notes but, at the same time, lose some details. In view of the fact that note recognition requires detailed information, the deep convolution layer feature information and shallower information are combined in this paper to obtain a feature map containing rich information, which enhances the model's learning ability for detailed features and improves the model's subsequent recognition ability. The feature extraction network combining multiscale feature fusion and residual CNN can effectively reduce the symbol error rate of the model and solve the problem of model nonconvergence. In training, serialized data requires forced alignment of data and label information. In the process of dealing with such problems, the combination of RNN and CTC has good performance, which constitutes different path probabilities by selecting notes and maximizes the path probability as an optimization goal. As a variant of RNN, the calculation of the gate state of SRU has nothing to do with the information output at the previous moment, so it can increase the amount of parallel calculation and accelerate the convergence speed of the model by solving the dependence of long-distance information. To fully exploit the locally consistent structure within the modalities of multimodal data, a cross-modal retrieval method fused with graph convolution is proposed. We utilize a symmetric graph convolutional encoding network and a symmetric multilayer fully connected encoding network to encode the raw features of samples from different modalities. The different encoded features are fused into a common representation learning layer shared by the input weights. This paper analyzes the experimental effect of the algorithm, including the influence of the number of iterations and the number of neurons in the hidden layer on the experiment. In addition, in order to illustrate the accuracy and rationality of the algorithm, the generated music sequence spectrograms are analyzed. At the same time, a comparative experiment was carried out to compare the spectrograms of the original music sequence and the cross-media audio and video score sequence. It can be found that the error of the experiment is very small through the spectrogram. Before performing the spectrogram analysis, the generated music sequence is also subjected to signal framing processing, and the processed music is generating a spectrogram. To illustrate that different genres of music can be generated, this chapter also presents the classification results of the generated music, which illustrate the conclusion through the classification results. In addition, in order to supplement the integrity of the experiment, the comparison between the traditional music generation algorithm and the algorithm proposed in this paper is also verified, which shows that the accuracy of the algorithm based on the convolutional neural network model in this paper is better than the traditional cross-sectional algorithm.

## Figures and Tables

**Figure 1:** Schematic diagram of multiscale feature fusion.

**Figure 2:** Building a modal diagram.

**Figure 3:** The effect of different iterations on the training effect.

**Figure 4:** Different effects of different iterations on the music spectrogram of the same song.

**Figure 5:** The effect of the number of neurons in the hidden layer on the error. Spectrogram analysis of cross-media audio and video score sequences.

**Figure 6:** Spectrogram of speech under different hidden layers.

**Figure 7:** Algorithm accuracy in genre classification.

**Figure 8:** Classification results of cross-media audio and video scores.

**Figure 9:** Comparison of the RBM cross-media audio and video score spectrogram with the music spectrogram in this paper.

## Data Availability

The data used to support the findings of this study are available from the corresponding author upon request.
